This article has been retracted.

# Evaluation Model of Physical Education Effect: On the Application of Radial Basis Function-Particle Swarm Optimization Neural Network (RBFNN-PSO)

**DOI:** 10.1155/2021/6819493

**Published:** 2021-07-30

**Authors:** Dong Chen

**Affiliations:** Sports Culture Research Base, Nanjing University of Information Science & Technology, Nanjing 210044, Jiangsu, China

## Abstract

This study constructs a new radial basis function-particle swarm optimization neural network (RBFNN-PSO) system, which is applied to the evaluation system of physical education teaching effect. In order to verify the evaluation performance of the RBFNN-PSO system, the traditional RBF neural network system is used as the control, and the training is carried out. The results show that the RBFNN-PSO system can reach the convergence value faster than the traditional RBF neural network system in the training, and the training error is smaller. The results show that the scoring error of RBFNN-PSO system is smaller than that of RBF neural network system, with higher accuracy and smaller error. The experimental results show that the RBFNN-PSO is superior to the traditional RBF neural network in error and accuracy.

## 1. Introduction

The evaluation of the teaching effect of curriculum is not only the evaluation of the teaching process and effect of the teacher, but also the assessment of the students' learning effect. The evaluation of teaching effect has become a powerful guarantee for the quality of curriculum teaching and an effective method to understand the quality of classroom teaching. At present, many students still use the traditional evaluation mode in teaching quality evaluation, with limited content, less times of assessment, and low data coverage, the students' learning quality problems cannot be reflected truthfully and completely, and teachers cannot find the problems and short boards in the teaching process in time. In order to improve the teaching quality, it is urgent to establish a scientific evaluation system of teaching effect [1].

In recent years, the research of teaching system has made some achievements. Elamrousy et al. [2] have made effective evaluation on the teaching performance of teachers in some educational courses. This study uses the method of analysis and description and compiles a questionnaire to evaluate the teaching performance of the staff. The results show that there is no statistical significance in the evaluation of the performance of some teaching staff in the education course in terms of age and professional degree, but there are differences in the evaluation and feedback methods for older students. There are also some achievements in the research of using intelligent algorithm to improve the accuracy of teaching evaluation. Liu et al. [3] put forward a new approach model which uses radial basis function to establish objective function and constraint for solving the problem of multiobjective optimization. The effectiveness and practicability of the method are verified by two numerical examples and two engineering examples. Because of the lack of global optimization ability in neural network method, it is necessary to optimize. Li et al. [4] put forward a combination of model and *k*-means++ method to optimize the key parameters of clustering, which provides a new method for text clustering. Shuai et al. [5] proposed a personal credit evaluation method based on RBFNN-PSO. The algorithm is used to optimize the parameters of RBFNN-PSO system, and the global search ability of RBFNN-PSO system and the efficiency of local optimization of RBFNN-PSO system are combined to overcome the instability of the algorithm and the disadvantage that algorithm can easily lead to local minimum. It has high accuracy in classification and prediction.

Neural network system for teaching effect evaluation has achieved certain results; through the comparison and research of various neural network algorithms, this study selects RBF algorithm to evaluate the effect of physical education teaching. The hidden node of traditional BP neural network uses the inner product of input pattern and weight vector as the independent variable of activation function, and each tuning parameter has the same influence on the output of the network. The hidden node of RBFNN-PSO system uses the distance between the input pattern and the central vector (such as Euclidean distance) as the independent variable of the function. The farther the input of the neuron is from the center of the radial basis function, the lower the activation degree of the neuron. BP neural network is the global approximation of nonlinear mapping. The output of RBFNN-PSO system is related to some tuning parameters, so RBFNN-PSO system has the characteristic of “local mapping.” There are many types of information in the evaluation of teaching effect, and all kinds of information have different degrees of influence on the teaching effect. Local mapping can more accurately reflect the internal relationship between these influences. The innovation of this research is to improve the traditional algorithm by RBFNN-PSO algorithm and build a new RBFNN-PSO system model. The performance of traditional RBF model depends on the selection of parameters to a large extent, while some parameters need to be optimized in the later stage for specific samples. The model only needs to assign the RBFNN-PSO algorithm, then the optimal parameters needed by the model can be obtained by using the excellent optimization ability of RBFNN-PSO algorithm, and the performance of the system can be improved.

This study is mainly of four parts.  Section 1 is the establishment of RBFNN-PSO system and the determination of the parameters with optimization.  Section 2 is the optimization of parameters of RBF model by RBFNN-PSO algorithm, and the evaluation system of teaching effect of RBFNN-PSO system is established.  Section 3 is the training results and the actual results of the RBFNN-PSO teaching effect evaluation system.  Section 4 summarizes the experimental results and summarizes the whole paper.

### 1.1. Establishment of RBFNN-PSO System

RBFNN-PSO system is essentially a special BP (back propagation) neural network [6]. From the structure, RBF neural network can be divided into three layers, namely the input layer of the first layer, the hidden layer of the second layer, and the output layer of the third layer. The overall structure is relatively simple. The input layer of the second layer is composed of sample input nodes; that is, after sample input, it will directly enter the hidden layer from the input layer. It can be understood that the hidden layer is the weighted average of each weight value equal to 1 between neurons in the input layer [7]. The hidden layer neuron uses Gaussian radial basis function *g*(*x*) as the excitation function, the output layer is the linear weighted average of the hidden layer, and the weight is set as *w*. The structure of RBF neural network is shown in Figure 1.

As shown in Figure 1, radial basis function is a kind of scalar function with radial symmetry, which is usually defined by Euclidean distance as follows:

(1) $$\begin{array}{c} \Phi_{i}\left(x\right)=G\left(\frac{\left\|x-c_{i}\right\|}{\sigma_{i}}\right). \end{array}$$

The commonly used Gaussian radial basis functions are shown in

(2) $$\begin{array}{c} \Phi_{i}\left(x\right)=\exp\left(-\frac{{\left\|x-c_{i}\right\|}^{2}}{2\sigma_{i}{}^{2}}\right). \end{array}$$

In (1) and (2), Φ_*i*_(*x*) is the output result of radial basis function, *x* is the input sample vector, *c*_*i*_ is the core of Gaussian radial basis function, and *σ*_*i*_ is the width of Gaussian radial basis function, representing the selectivity of neurons [8]. When the center *c* is equal to 0 and the width *σ* is 1, the function graph is shown in Figure 2.

It can be seen from Figure 2 that the closer *x* value is to the center *c*, the closer the function value is to the peak value. When the width *σ* is larger, the graph of the function is wider and the response range of *x* is correspondingly larger. On the contrary, when the width *σ* is smaller, the graph of the function is narrower, and the response range of *x* is correspondingly smaller [9]. Only samples close enough to the center can activate neurons, so only some neurons in the hidden layer contribute to the output. When the input value *x* is *p* dimension and the output value (set as *y*) is *k* dimension, the expression formula of RBF network can be expressed as

(3) $$\begin{array}{c} y_{k}=\Phi_{i}\left(x_{k}\right)=\sum_{i=1}^{m}w_{ik}\exp\left(-\frac{{\left\|x_{p}-c_{i}\right\|}^{2}}{2\sigma_{i}{}^{2}}\right). \end{array}$$

It can be seen from (3) that RBF neural network algorithm can be used for local approximation of nonlinear functions. In each approximation operation, only part of the parameters is called, so the amount of calculation is greatly reduced and the operation speed is improved. RBF neural network algorithm needs to preprocess the samples, usually do clustering processing, in order to ensure the selectivity of the algorithm, and process large samples or multifeature samples more quickly and accurately [10]. The radial function of hidden layer of RBF neural network can segment high-dimensional nonseparable data into low dimensional separable linear data by interpolation. RBF neural network full-interpolation method is divided into Lagrange interpolation, Hermite interpolation, Newton interpolation, spline interpolation, piecewise interpolation, and so on [11]. The interpolation function of complete interpolation method needs to pass through all sample points, and the formula expression is as follows:

(4) $$\begin{array}{c} F\left(x_{m}\right)=Y_{m}. \end{array}$$

In (4), *x*_*m*_ is *m* 1 × and *M* > *n*; *Y*_*m*_ is the corresponding output of *x*_*m*_. A RBF neural network with *m* centers is constructed, and the Gaussian radial basis function is selected as the hidden layer activation function. The structural equations of the function are shown in (4).

(5) $$\begin{array}{c} \left\{\begin{array}{c} w_{1}G\left(\left\|x_{1}-c_{1}\right\|\right)+w_{2}G\left(\left\|x_{1}-c_{2}\right\|\right)+\ldots +w_{m}G\left(\left\|x_{1}-c_{m}\right\|\right)=Y_{1},\\ w_{1}G\left(\left\|x_{2}-c_{1}\right\|\right)+w_{2}G\left(\left\|x_{2}-c_{2}\right\|\right)+\ldots +w_{m}G\left(\left\|x_{2}-c_{m}\right\|\right)=Y_{2},\\ \vdots \\ w_{1}G\left(\left\|x_{m}-c_{1}\right\|\right)+w_{2}G\left(\left\|x_{m}-c_{2}\right\|\right)+\ldots +w_{m}G\left(\left\|x_{m}-c_{m}\right\|\right)=Y_{m}. \end{array}\right) \end{array}$$

In (5), center *c*=[*c*_1_, *c*_2_,…, *c*_*m*_], input *x*=[*x*_1_, *x*_2_,…, *x*_*m*_], hidden layer *G*=[*G*(‖*x* − *c*_1_‖), *G*(‖*x* − *c*_2_‖),…,*G*(‖*x* − *c*_*m*_‖)]^*T*^, weight *w*=[*w*_1_, *w*_2_,…, *w*_*m*_], and output *Y*=[*Y*_1_, *Y*_2_,…, *Y*_*m*_]. In (5), the input matrix and the matrix are transformed into *M* × *M* matrix, and the mapping from low dimension to high dimension is realized [12]. Formula (5) is expressed in the form of vector, such as

(6) $$\begin{array}{c} Gw^{T}=Y^{T}. \end{array}$$

Formula (6) shows that the matrix *G* is invertible when the hidden layer kernel function is Gaussian radial basis function. After multiplying the left and right sides of (6) by G − 1 at the same time, we transpose the matrix to get

(7) $$\begin{array}{c} w={\left(G^{-1}Y^{T}\right)}^{T}. \end{array}$$

Transpose formula (7) again to get formula (8).

(8) $$\begin{array}{c} G\left(x,c\right)w^{T}=Y^{T}. \end{array}$$

Formula (8) is the complete interpolation function of RBF neural network. *C* in the formula can be set randomly. It can be seen from formula (8) that as long as the parameters of the hidden layer kernel function are determined, the interpolation function can be uniquely determined. This shows that RBF neural network can completely interpolate and fit any nonlinear function [13]. Next, select the data points, and use RBF neural network to carry out one-dimensional fitting and exponential fitting for the data. See Figure 3 for the graph.

In Figure 3, the number of RBF neural network centers is set to 10, and the input values are evenly distributed along the *x*-axis. The hidden layer of RBF is obtained, and the result is shown in the red curve in Figure 3(b). Select a data point (set as point *a*) on the left side of *x*-axis in Figure 3(b) for fitting. The *f* (*x*) value of *a* corresponds to the linear weighting of all central kernel functions corresponding to *x*1. The fitting method of other data points is the same as that of point *a*. As can be seen from Figure 3(c), only the two hidden layer kernels on the far left contribute to *x*1; that is, the hidden layer kernels in the width range of *X*1 contribute to *x*1, and the kernels far away from its center contributing to the output of *X*1 are all 0. From the process of fitting, we can see that the center, width, and weight determine the output of RBF neural network, which can be understood as the training process of RBF neural network. In essence, it is the process of optimizing these three parameters.

### 1.2. Parameter Setting of Model

In order to make an objective and correct evaluation of teaching quality, it is necessary to establish an evaluation system of physical education teaching effect. The evaluation system of teaching effect established in this study is divided into two levels, each level is given a weight. The specific evaluation items are shown in Table 1.

The results of each item in Table 1 can be divided into four grades: “excellent”, “good”, “medium”, and “poor”, which are expressed by *a*, *B*, *C,* and *D,* respectively. *X*_*ij*_ is used to represent the frequency of each level of evaluation, *W*_*ij*_ is used to represent the weight of each evaluation item.

(9) $$\begin{array}{c} A=\left\{\begin{array}{cccc} X_{11A} & X_{11B} & X_{11C} & X_{11D}\\ X_{12A} & X_{12B} & X_{12C} & X_{12D}\\ \vdots & \; & \; & \;\\ X_{mnA} & X_{mnB} & X_{mnC} & X_{mnD} \end{array}\right\}. \end{array}$$

In (9), the weight functions of *i*=1,2,…, *m*, *j*=1,2,…, *n*, and the weight function are shown in

(10) $$\begin{array}{c} W=\left\{\begin{array}{cccc} W_{11} & W_{12} & \cdots & W_{1j}\\ W_{21} & W_{22} & \cdots & W_{2j}\\ \vdots & \; & \; & \;\\ W_{i1} & W_{i2} & \cdots & W_{ij} \end{array}\right\}. \end{array}$$

The quality level can be expressed as

(11) $$\begin{array}{c} Q=\left(Q_{A},Q_{B},Q_{C},Q_{D}\right). \end{array}$$

*Q*_*A*_, *Q*_*B*_, *Q*_*C*_, and *Q*_*D*_ in the quality level can be assigned to 1, 2, 3, and 4, respectively, in this experiment. Input the sample data and output the result of teaching quality evaluation. In the actual operation process, the parameters need to be initially set and optimized before inputting samples [14, 15]. In theory, the number of centers should be equal to the number of sample categories. At the same time, each sample is required to have a good distinction and independence. At the same time, each sample is required to have a probability distribution model around the center and obey a model similar to radial basis function. These two requirements are difficult to achieve (width parameter *σ*). The optimization idea of the weight parameter *W* is similar to that of the central parameter, which should be further solved in the later training process. In this study, algorithm is used to optimize it, and an improved RBFNN-PSO system is constructed.

## 2. Establishment of Physical Education Teaching Effect Evaluation System Based on RBFNN-PSO System

### 2.1. Construction of RBFNN-PSO System

RBFNN-PSO system is based on RBF neural network, and the parameters in RBFNN-PSO system are optimized by using PSO (particle swarm optimization) algorithm. Width parameter *σ*, the weight parameter *w*, and the center parameter *c* need to be optimized by algorithm. Firstly, a target search space needs to be set. *M* vectors form a collection. Each particle in the collection has *n*-dimensional eigenvalues. The current position of the first particle in the collection is recorded as *p*_*i*_. *p*_*i*_ is substituted into the target function to get an output value. When the output does not meet the algorithm termination requirements, the position will be updated and moved to *p*_*i*+1_. The formula of particle displacement update is

(12) $$\begin{array}{c} p_{i+1}=p_{i}+\alpha \nu_{i}. \end{array}$$

In (12), *p*_*i*+1_ is the updated position of particle *m*, *p*_*i*_ is the current position of particle *m*, *α* is the flight time of particle, and *ν*_*i*_ is the current flight speed of particle. There are three main factors influencing the update of particle flight speed *ν*_*i*_: the flight inertia of the particle at the last moment, individual flight experience, and global flight experience [16]. In order to prevent the particle velocity from being too large or too small, resulting in no displacement after updating, it is necessary to add a certain limit to the flight velocity *ν*_*i*_ of the particle in the flight process, such as *ν*_*i*_ ∈ [*v*_min_, *v*_max_], where *v*_min_=−*v*_max_, when *ν*_*i*_ < *v*_min_ or *ν*_*i*_ > *v*_max_ occurs. Then *ν*_*i*_=*v*_min_ or *vi*+1=*wvi*+*c*1*r*1(*p*best − *pi*)+*c*2*r*2(*g*best − pi) [17]. The particle displacement update formula can be expressed as

(13) $$\begin{array}{c} v_{i+1}=wv_{i}+c_{1}r_{1}\left(p\text{best}-p_{i}\right)+c_{2}r_{2}\left(g\text{best}-p_{i}\right). \end{array}$$

In (13), *w* represents inertia factor, *c*_1_ represents individual accelerated learning factor, *c*_2_ represents global accelerated learning factor, *r*_1_ and *r*_2_ represent random numbers in the range of [0, 1], *p*best represents local optimal position, and *g*best represents global optimal position [18]. The termination condition of algorithm iteration is set according to the specific problem, which can set the maximum number of iteration steps, or the error can meet the requirements. The specific algorithm flow is shown in Figure 4.

As can be seen from Figure 4, the operation flow of PSO algorithm is mainly as follows. STEP. 1: initial particle number setting, the initial position and velocity of particles are set. The parameters of inertia factor and accelerated learning factor are set. Set the iteration termination condition, which can be the maximum number of iterations or the minimum error requirement [19]. STEP. 2: the output value of the objective function of the initial position of each particle is calculated, and the corresponding error is calculated. STEP. 3 : The position Pi of the initial point of each particle is denoted as pbest, the position of the initial point of the particle with the least mean square error of the initial points of all particles is selected, and the position is denoted as gbest. STEP. 4 : Update the current position and velocity of each particle according to formulas (12) and (13). STEP.5 :  the output value and error of each particle after updating its position are calculated. STEP. 6 : judge whether the iteration termination condition is satisfied. If the condition is satisfied, go to Step 9, if not, the current position error of each particle is compared with the pbest position error of the particle. In case of Gbest point error, go to Step 7. STEP. 7 : when the current position error of a particle is less than the *p*best position error of the particle, the current position of the particle is updated to *p*best. STEP. 8 : if the minimum error of the current position of all particles is less than the error of the previous gbest position, the pI value of the minimum error of the current particle position is updated to *g*best, and return to Step 4. STEP. 9 : at the end of the iteration, the gbest vector of the global optimal solution is obtained [20].

It can be seen from the operation process that the setting of parameters in PSO algorithm has a great impact on the performance of the algorithm. The main influence parameters are particle number *m*, inertia factor *w*, maximum flight speed *v*_max_, individual accelerated learning factor *c*_1_, and global accelerated learning factor *c*_2_ [21]. The number of particles *M* will determine the number of potential solutions of PSO algorithm. The larger the number of particles *M* is, the stronger the optimization ability of PSO algorithm is, and the corresponding amount of computation in each iteration will increase [22]. By consulting the data, we can see that, for the general scale problem, the number of particles *m* is 20 to 40. The inertia factor *w* can determine the inheritance degree of the algorithm to the original speed and path direction. The larger the inertia factor *w* is, the greater the flight inertia of the particle is. When the particle deviates from the original path in flight, the smaller the inertia factor *w* is, it is conducive to local optimization, and the global optimization ability is weakened [23–25]. In the actual operation process, there will be different operation stages and different requirements for the global search ability. For example, in the early stage of operation, we hope the algorithm has strong global search ability, and in the later stage, we hope the algorithm has strong local optimization ability [26–28]. We can adjust the value of inertia factor *w*. The adjustment method is shown in (14) and (15).

(14) $$\begin{array}{c} w=w_{\max}-\frac{k\times \left(w_{\max}-w_{\min}\right)}{k_{\max}}, \end{array}$$

(15) $$\begin{array}{c} w=w_{\max}-\frac{\mathrm{lg}\left(k\right)}{\mathrm{lg}\left(k_{\max}\right)}\times \left(w_{\max}-w_{\min}\right). \end{array}$$

In (14) and (15), *w*_max_ is the maximum inertia factor, *w*_min_ is the minimum inertia factor, *k* is the current iteration number, and *k*_max_ is the maximum iteration number. Formula (14) is the dynamic adjustment formula of linear inertial factor, and formula (15) is the dynamic adjustment method of exponential inertial factor. The change of *w* value with the number of iterations is shown in Figure 5.

As can be seen from Figure 5(a), the linear adjustment formula of inertia factor *w* realizes the dynamic adjustment of inertia factor. In an ideal optimization process, the transition from global search to local search should be nonlinear, and the global search should be completed quickly. The exponential adjustment formula optimizes the linear adjustment formula, and the exponential curve of Figure 5(b) is more in line with the ideal optimization concept. There are adaptive method and random method to adjust the inertia factor, each of which has its own advantages and disadvantages. Through the data access method, combined with (14) and (15), the maximum velocity *v*_max_ of flying particles is set to 10% to 20% of each dimensional variable. To sum up, the number of particles *m* = 30, and the inertia factor *w* adopts the exponential dynamic inertia factor. Set *w*_max_=0.95, *w*_min_=0.4, the maximum flight velocity *v*_max_ is set to 0.6, the individual accelerated learning factor *c*_1_ is set to 2.04, and the global accelerated learning factor *c*_2_ is set to 2.04. The optimized parameters are used to establish RBF neural network. The establishment of RBFNN-PSO system is completed.

### 2.2. Construction of Teaching Effect Evaluation System

The data source of the teaching effect evaluation system is determined firstly. The data of the teaching effect evaluation system are from the 2019 teachers and students and some experts of the computer school of a university in Anhui Province. The database model contains the entity objects and corresponding data in 2019. The relationship is shown in Figure 6.

Figure 6 is the entity relationship diagram (*E*-*R* diagram) of the system data, mainly including departments, majors, and classes, as well as members, students, experts, peer teachers, teachers, etc., which are connected through physical education curriculum [29, 30]. Physical education curriculum is a specific form of teaching activities, physical education teachers through physical education curriculum and students teaching relationship. There are logical relations between all kinds of entity objects, such that the relationship between department objects and professional objects is one to many, the logical relationship between students and physical education teachers is many to one, and the logical relationship between experts and peer teachers and physical education teachers is many to many. In the evaluation system, the evaluation data need to enter the database in the server and then access multiple servers through the network card and gateway. The network structure of the evaluation system is shown in Figure 7.

In Figure 7, a service program is configured on the web server to configure the evaluation data to the corresponding server database. The mobile phone client and the computer client can access the server data simultaneously through the network card and the internal gateway, and the external network can be accessed through the LAN device in the router. In order to prevent external network attacks, the evaluation system also set up an external firewall. The construction of physical education teaching evaluation system is completed.

## 3. Experimental Results of RBFNN-PSO System

### 3.1. Training Performance Verification of RBFNN-PSO System

In this training, the questionnaire of 2019 grade teachers and students and some experts in the Computer College of a university in Anhui Province was extracted as the training data. In order to verify the superiority of the training effect, in addition to the RBFNN-PSO system, the traditional RBF neural network system is designed to train synchronously. The training data include 1000 student questionnaires, 100 peer and expert questionnaires, which constitute the training database. During the training process, 100 questionnaires were randomly selected from the database as training samples to train the two kinds of neural systems respectively. The error of the two neural network systems in the training process is shown in Figure 8.

It can be seen from Figure 8 that the error of the RBFNN-PSO system in the training process decreases significantly in the iterative process. After the number of iterations approaches 120, the error tends to be stable, and the error size is about 0.002. The error of RBF neural network system also decreases in the iterative process, but the decline process is relatively slow. The error gradually tends to be stable at about 200 iterations, and the stable error is about 0.005, which is about 2.5 times of the training error of RBFNN-PSO system. It shows that the training error of RBFNN-PSO system is smaller than that of traditional RBF neural network system, and it tends to be stable faster and reaches the convergence value faster.

### 3.2. Experimental Results of Trained RBFNN-PSO System

In this experiment, 200 groups of students' evaluation data were selected from the database and randomly divided into 4 groups. According to the effect of physical education teaching, the trained RBFNN-PSO system and the trained traditional RBF neural network system were used for the control experiment in the same experimental environment. The experimental results are shown in Figure 9.

 It can be seen from Figure 9 that in the four groups of experiments, there is a certain error between the scores obtained by the trained RBFNN-PSO system and the students' scores, and the absolute error is not more than 0.03. There is a certain error between the score of the trained traditional RBF neural network system and that of the students, and the absolute error is not more than 0.06. The score error of the traditional RBF neural network system is about twice that of the RBFNN-PSO system, which is basically consistent with the error of the training results. By randomly selecting 20 evaluation results of experts and peer teachers and taking the evaluation results of experts and peer teachers as the reference standard, the accuracy of the system scoring results can be verified. The experimental results are shown in Figure 10.

It can be seen from Figure 10 that the expert evaluation results are taken as the evaluation standard values, and the results of the trained RBFNN-PSO evaluation system are relatively close to the standard values at each data point, and the data points with an error of less than 5% account for 86%. The traditional RBF neural network system scoring results are basically consistent with the trend of the standard values, and the data points with an error of less than 5% account for 63%. Therefore, it can be proved that RBFNN-PSO system has significant advantages over traditional RBF neural network in performance. The error of RBFNN-PSO system is extracted and analyzed, and Figure 11 is obtained.

As can be seen from Figure 11, the scoring error of the RBFNN-PSO evaluation system is between −0.04, 0.04, and the error of most data points is controlled within the allowable range −0.02, 0.02, which proves that the system runs stably, and outliers appear in some extreme scoring data groups. The possible reason is that there are few training data for this kind of scoring and the error is relatively large. Therefore, the evaluation system is feasible in performance and stability.

## 4. Conclusion

This study optimizes the traditional RBF algorithm, uses the optimization ability of PSO algorithm, constructs a new RBFNN-PSO system, and integrates the system with the physical education teaching effect evaluation system. In order to verify the evaluation performance of the RBFNN-PSO system, the traditional RBF neural network system is used as the control, and the training is carried out. The results show that the RBFNN-PSO system can reach the convergence value faster than the traditional RBF neural network system in the training, and the training error is smaller. The results show that the error of RBFNN-PSO system is smaller than that of RBF neural network system, the accuracy is 23% higher, and the error is 50% lower. The experimental results show that the RBFNN-PSO is superior to the traditional RBF neural network in error and accuracy.

## Figures and Tables

**Figure 1:** RBFNN-PSO system structure diagram.

**Figure 2:** Gauss radial basis function diagram.

**Figure 3:** One-dimensional fitting of RBFNN-PSO. (a) Distribution of sample points. (b) Hidden layer kernel function distribution. (c) Point a data fitting.

**Figure 4:** Flow chart of RBFNN-PSO system algorithm.

**Figure 5:** Dynamic curves of two inertial factors. (a) Dynamic curve of linear inertia factor. (b) Dynamic curve of exponential inertia factor.

**Figure 6:** *E*-*R* diagram of the whole system.

**Figure 7:** Network architecture of evaluation system.

**Figure 8:** Two kinds of neural network training error.

**Figure 9:** Comparison chart of student scoring and system scoring results. (a) Group 1. (b) Group 2. (c) Group 3. (d) Group 4.

**Figure 10:** Comparison chart of system score and expert score.

**Figure 11:** System scoring error chart.

**Table 1:** Evaluation items of physical education teaching effect.

Evaluation index level 1		Weight (*W*_*i*_)	Evaluation index level 2	Weight (*W*_*ij*_)

1	Content of courses	*W*_1_	(1) The teaching is simple and easy to understand	*W*_11_
			(2) The key points and difficulties are prominent	*W*_12_
			(3) Finish teaching task on time	*W*_13_
			(4) The teaching content is rich and substantial	*W*_14_

2	Teaching attitude	*W*_2_	(1) Positive attitude and enthusiasm	*W*_21_
			(2) Prepare lessons actively and fully	*W*_22_

3	Teaching method	*W*_3_	(1) The lecture is easy to understand	*W*_31_
			(2) The key points and difficulties are prominent	*W*_32_
			(3) Finish teaching task on time	*W*_33_

4	Teaching effectiveness	*W*_4_	(1) Good communication between teachers and students	*W*_41_
			(2) Students master the sports skills they have learned	*W*_42_
			(3) Students get physical and mental exercise	*W*_43_
			(4) The students' interest in physical education is improved	*W*_44_

## Data Availability

The data used to support the findings of this study are available from the corresponding author upon request.
